# Effect and Clinical Value of Protective Motivation Intervention Rehabilitation Model on Pain Perception and Dysfunction in Patients with Lumbar Disc Herniation: Based on a Retrospective Cohort Study

**DOI:** 10.1155/2022/5911889

**Published:** 2022-08-30

**Authors:** Xingbang Liu, Yong He

**Affiliations:** ^1^Qianjiang Central Hospital, Hubei Province Qianjiang Hospital, People's Hospital of Wuhan University, Department of Orthopaedics, Qianjiang Clinical Medical College, Yangtze River University, China; ^2^Department of Orthopedics, Hubei Provincial Hospital of Traditional Chinese Medicine, China

## Abstract

**Objective:**

To examine the potential medical benefits of protective motivation intervention rehabilitation mode on pain perception and dysfunction in patients with lumbar disc herniation (LDH).

**Methods:**

140 LDH patients hospitalized from January 2021 to September 2021 were totally selected. The control group received regular rehabilitation, and the research group received protective motivation intervention rehabilitation. The comparisons of scores of disease knowledge, visual analogue scale (VAS), pain belief and perception scale (PBPI), Japanese Orthopedic Association Score (JOA), Roland-Morris dysfunction (RMDQ), and quality of life scale (SF-36) were made across different groups.

**Results:**

The scores of disease knowledge in the two cohorts at 1 month, 2 months, and 3 months after intervention were greater than those before intervention, and the difference is statistically significant (*P* < 0.05). The scores of VAS, PBPI, JOA, and RMDQ at 1 month, 2 months, and 3 months after intervention were downregulated. At 1 month, 2 months, and 3 months after intervention, the experimental scores of VAS, PBPI, JOA, and RMDQ were markedly fewer than the control group, and the difference is statistically significant (*P* < 0.05). The scores of SF-36 after intervention were statistically upregulated, and the difference is statistically significant (*P* < 0.05). After intervention, the score of SF-36 in the research group was significantly higher than that in the control group, and the difference is statistically significant (*P* < 0.05).

**Conclusion:**

The application of protective motivation intervention in rehabilitation of LDH patients can more effectively improve their cognitive level, reduce their pain perception, improve their lumbar function, and enhance their well-being.

## 1. Introduction

Lumbar disc herniation (LDH) is a phenomenon in which degenerative alterations occur in various parts of the lumbar disc, resulting in rupture of the fibrous ring and protrusion of the nucleus pulposus tissue from the rupture, thereby irritating or compressing the spinal nerve roots and presenting a range of symptoms [1–3]. The current research has displayed that the incidence of LDH in western countries is 15.2% MUE 30%. The incidence of LDH in China has reached 15.2% [4]. The main population is young and middle-aged adults with an average age of about 40 years old. Most of them are drivers, heavy manual workers, and sitting/learning-based workers [5]. The incidence of male patients is significantly higher than female, which may be related to men that are normally engaged in high-intensity and high-load work. The recent study has suggested that with the improvement of education, the risk of LDH decreases. The vast majority of LDH patients are always suffering from back pain and often a range of functional impairments. The patients usually experience both physical pain and heavy psychological burden, resulting in a severely reduced quality of life [6, 7]. Therefore, reducing pain and enhancing well-being of LDH patients has become a priority for clinical nurses.

Generally, 10%-18% of LDH patients need surgical treatment, and 80% of patients can be cured by surgery. This is mainly because surgery can be a direct, quick, and effective way to remove the discs that produce nerve compression [8]. However, surgical treatment is an invasive operation and can result in postoperative complications. The related literature has reported that about 30% of the patients had primary or secondary low back pain, 20% of the patients had residual leg pain, and 30% of the patients had significantly reduced flexibility of the lumbar spine [9, 10]. Earlier rehabilitation after operation can obviously shorten the rehabilitation time, reduce postoperative complications, and improve cardiopulmonary function. Currently, the relatively conservative view is that early postoperative functional exercise can affect the internal fixation and lead to loosening of the fixation or even fracture [11]. It is suggested that bone healing can be achieved by fixation and interbody fusion within 3 months after operation. Functional rehabilitation training should be carried out to reduce the risk of internal loosening. The protection motivation theory (PMT) was first put forward and gradually developed by American scholar Rogers in 1975, which belonged to the theory of healthy psychology. The theory suggests that behaviors and attitudes can be changed through a process of cognitive regulation, emphasizing the importance of inherent cognition in the decision-making process of health behaviors. It is also considered that a series of cognitive processes in which environmental factors affect behavior can be explained by two assessment approaches, including threat assessment and coping assessment [12]. A threat assessment is an individual's understanding of unhealthy behavior, which is formed by balancing the perceived benefits and risks associated with adopting risky behaviors. Coping assessment is the individual's understanding of his own ability to deal with unhealthy behavior, and it is the judgment formed by the individual after comprehensively comparing the effective perception of behavior change, the confidence of changing unhealthy behavior, and the obstacles encountered in the process of behavior change [13, 14]. The protective motivational intervention model allows for better patient motivation, increased patient awareness of the disease, and improved patient-related behaviors through psychological regulation and aspects of daily living. Therefore, this study explored the effect and clinical value of protective motivation intervention rehabilitation model on pain perception and dysfunction in patients with LDH.

## 2. Materials and Methods

### 2.1. General Information

A total of 140 patients with LDH hospitalized from January 2021 to September 2021 were selected as the research objects. All cases were divided into the control group and the research group by random number table method. The control group was implemented routine rehabilitation and the research group was implemented protective motivation intervention rehabilitation. The age of control group ranged from 31 to 74 years old with an average age of 34.53 ± 3.52 years, including 42 males and 28 females. The age of research group ranged from 31 to 73 years with a mean age of 33.92 ± 3.41 years, including 40 males and 30 females. There was no significant difference in general data between the two groups (*P* > 0.05). All patients signed informed consent before this study. This study was a double-blind test.

Inclusion criteria are as follows: (1) patients with LDH diagnosed by CT or MRI with stable condition; (2) age > 18 years; (3) clear consciousness, basic reading, and writing ability; (4) language communication barrier-free; and (5) the patients agreed to participate in this researcher.

Exclusion criteria are as follows: (1) severe lumbar spinal stenosis caused by LDH combined with lumbar spondylolisthesis and hyperosteogeny; (2) pathological bone fracture history and neuromuscular system diseases associated with severe osteoporosis; (3) patients with previous history of mental illness and cognitive impairment or suspected cognitive impairment before brain trauma; (4) patients with myocardial infarction or with severe liver and kidney dysfunction, severe infection, severe diabetes, etc.; (5) missing follow-up; (6) patients voluntarily asked to withdraw from the study; and (7) serious morbidity or death occurred in the course of the study.

### 2.2. Methods

The control group accepted routine rehabilitation. During the period of hospitalization, routine rehabilitation nursing services were carried out, such as life intervention, diet intervention, psychological intervention, treatment cooperation guidance, disease knowledge publicity and education, exercise guidance, and telling patients to stay in bed.

The research group accepted protective motivation to intervene rehabilitation model. The intervention rehabilitation program was made according to seven factors of protective motivation, namely, internal return, severity, self-efficacy, response efficacy, susceptibility, external return, and response cost. (1) Severity and susceptibility: patients have limited mastery of disease and surgery, which can easily lead to negative emotions such as anxiety, tension, and fear. Clinical nursing staff should give corresponding knowledge explanation in time and make good preparation before operation. Within 1 week after admission, centralized education was carried out for 3 times, each time for 30 minutes. The way of watching video and explanation was used to explain the causes, treatment methods, and prognostic factors of LDH and to explain in detail the matters needing attention in operation. Inform patients of the harm that bad lifestyle may bring and improve patients' attention to the disease. In addition, psychological counseling intervention should be given to different patients to comfort and encourage them to build up their confidence in treatment. (2) Internal and external returns: correction of patients' misconceptions and behaviors and weakening of internal reward factors (e.g., patients' poor lifestyle habits) and external reward factors (e.g., neglect of disease risk factors by family and friends) through experience sharing sessions and individual coaching. Following your doctor's advice was highlighted as a positive for improving your condition.

Assess the patient's psychological status and self-care ability and develop a personalized functional exercise program and promote the patient to cooperate with the treatment recommended by the doctor and obtain internal rewards according to the personalized plan. Strengthen the support of the patient's family by explaining relevant disease knowledge to increase the patient's sense of security and alleviate their adverse psychological emotions, which in turn will improve their confidence with surgical treatment. (3) Response efficacy and self-efficacy: through collective education and experience sharing, the patients' cognitive level of lumbar disc herniation was improved and patients' self-care ability was enhanced to help patients familiarize themselves with rehabilitation exercise methods after lumbar disc herniation. Patients are guided to adopt healthy self-intervention behaviors to improve self-intervention, enhance response to treatment, and improve their confidence in recovery. (4) Reaction cost: individual guidance was given to patients to help them understand the positive impact of health-related self-intervention on the prognosis of the disease. After patients are discharged from hospital, we continue to provide care through family follow-up visits and telephone follow-up. We continue to actively answer patient-related questions and encourage patients' families to monitor patient-related behaviors to maximize patient motivation. In addition, through follow-up and organizing patient communication meetings, we can help patients solve their daily difficulties and make them realize that the benefits of intervention and treatment are higher than their own psychological or disease reaction costs. The rehabilitation in both groups included professional physical therapy. The frequency and duration of each activity were the same in both groups. Both groups exercise 20 min each time, 4 times a day. Both groups were intervened continuously for 4 weeks.

### 2.3. Observation Index

#### 2.3.1. Disease Knowledge Score

The disease knowledge level was evaluated by the disease knowledge scale of lumbar disc herniation. The scale included exercise, disease, rehabilitation intervention, daily life, diet, and other evaluation items [15]. The total score was 34. The higher the score, the higher the cognitive level of patients' knowledge related to LDH.

#### 2.3.2. Pain Degree

Visual analogue scale (VAS) was used to evaluate the degree of pain [16]. The score of the VAS scale ranges from 0 to 10, in which “0” represents “painless” and “10” represents “unbearable pain”. 1-2 is for mild pain, 3-5 is for moderate pain, and more than 5 is for severe pain. The higher the score, the stronger the pain. The Cronbach's *α* coefficient of the questionnaire was 0.887.

#### 2.3.3. Pain Belief and Perception

The Pain Belief and Perception Inventory (PBPI) was used to evaluate the pain belief of patients, including four dimensions [17]: persistent pain, mysterious pain, irremediable pain, and self-blame with 16 entries. Using the 4-grade scoring system, the scores from “very disagree” to “very agree” were -2, -1, +l, and +2, respectively. The sum of all the items was the total score. The higher the score, the stronger the negative belief held by the patient. At present, the scale has been mainly used to evaluate patients with chronic pain in China. The Cronbach's *α* coefficient of each dimension is 0.735-0.883, and the Cronbach's *α* coefficient of the total scale is 0.731.

#### 2.3.4. Spinal Cord and Neurological Function

Japanese Orthopedic Association Score (JOA) was used to evaluate the spinal cord and nerve function [18]. The scale included subjective symptoms, clinical symptoms, and limitation of daily activities and bladder function. The highest total score of JOA was 29 and the lowest was 0. The higher the score, the better the spinal cord and nerve function.

#### 2.3.5. Lumbar Vertebra Dysfunction

The degree of lumbar dysfunction was evaluated by Roland-Morris Lumbar Disorder scale (RMDQ) [19]. The scale included 24 questions. The answer to “yes” obtained 1 point and the answer to “no” obtained 0. The total score of each item was the total score. The higher the total score, the more obvious the degree of lumbar dysfunction. The Cronbach's *α* coefficient of the scale is 0.83. Each question is limited by the phrase “due to low back pain,” including the effects of low back pain on walking, dressing, bending, sitting, lying position, sleep, self-care ability, and daily life.

#### 2.3.6. Quality of Life Scale

The life quality scale was evaluated by SF-36 health survey table [20]. 8 items were included, such as physiological function, psychological function, body painful feelings, common medical conditions, energy, social functioning, emotional functioning, and psychological well-being. The each dimension mark was from zero to one hundred.

### 2.4. Statistical Analysis

The statistical package SPSS 21.0 would be used to analyze the data. (s) was used to represent the measured data. The groups were compared using an independent sample *t*. Both during treatment, a paired *t*-test would be used to compare the two groups. Furthermore, number data was written as *n* (percent). The qualify data were compared using the *χ*^2^ test. The result differed when *P* < 0.05 was used.

## 3. Results

### 3.1. Comparison of Disease Knowledge Scores

No great differences were exhibited in the score of disease knowledge before intervention (*P* > 0.05). The disease knowledge in both groups at 1 month, 2 months, and 3 months after intervention was greatly larger than those prior intervention (*P* < 0.05). At 1 month, 2 months, and 3 months after intervention, the score of disease knowledge in the research group was obviously greater than that in the control group (*P* < 0.05). All results are shown in Table 1.

### 3.2. Comparison of Pain Degree

No obvious differences appeared in the score of VAS scale prior intervention. The patients in the experimental group had less pain during one-month, two-month, and three-month intervention (*P* < 0.05). All cases experienced a reduction in pain after the intervention (*P* < 0.05). All results are shown in Table 2.

### 3.3. Comparison of Pain Belief and Perception

Before intervention, there was no significant difference in PBPI scores between the two groups (*P* > 0.05). The PBPI scores of the two groups at 1 month, 2 months, and 3 months after intervention were significantly lower than those before intervention (*P* < 0.05). After 1 month, 2 months and 3 months after intervention, the PBPI score of the research group was lower than that of the control group with the statistically significant difference (*P* < 0.05). All results are shown in Table 3.

### 3.4. Comparison of Spinal Cord and Nerve Function

Before intervention, there was no significant difference in the JOA score between the two groups (*P* > 0.05). The JOA scores of the two groups at 1 month, 2 months, and 3 months after intervention were significantly lower than those before intervention (*P* < 0.05). After 1 month, 2 months, and 3 months after the intervention, the JOA scores of the research group were lower than those of the control group with the statistically significant difference (*P* < 0.05). All results are shown in Figure 1.

### 3.5. Comparison of Lumbar Disorder

Before intervention, there was no significant difference in the RMDQ scores between the two groups (*P* > 0.05). The RMDQ scores of the two groups at 1 month, 2 months, and 3 months after intervention were significantly lower than those before intervention (*P* < 0.05). After 1 month, 2 months, and 3 months after the intervention, the RMDQ scores of the research group were lower than those of the control group, and the difference was statistically significant (*P* < 0.05). All results are shown in Figure 2.

### 3.6. Comparison of Quality of Life

Before intervention, there was no significant difference in SF-36 scores between the two groups (*P* > 0.05). The SF-36 scores of the two groups after intervention were significantly higher than those before intervention (*P* < 0.05). After intervention, the SF-36 scores of the research group were larger than those of the control group, and the difference was statistically significant (*P* < 0.05). All results are shown in Table 4.

## 4. Discussion

With the continuous change of people's working environment and lifestyle, the incidence of LDH is increasing year by year. LDH has become a modern international epidemic disease [21, 22], which is harmful to human health. Therefore, it is of great practical significance to study the more beneficial rehabilitation treatment of LDH and to explore effective clinical treatment. At present, the methods for the treatment of LDH are divided into two categories, consisting of surgical treatment and nonoperative treatment [23, 24]. More and more clinical attention has been paid to the treatment of LDH with nonoperative therapy. According to relevant literature reports, about 80.00% of patients can be relieved or cured by corresponding nonoperative treatment. However, after the prolapse of lumbar intervertebral disc, the multifid muscle of many patients has obviously atrophied. With the extension of the course of the disease, the multifid muscle atrophy is becoming more and more serious, which leads to the poor effect of nonoperative treatment [25–27]. After surgical treatment, some patients can achieve good outcomes, but a few of studies have shown that patients with LDH are prone to postoperative complications, limited movement of lumbar vertebrae, and weakness of lower limbs, which can seriously affect normal work and life.

Previous studies have shown that perioperative rehabilitation therapy can be used as one of the effective means to prevent postoperative complications [28, 29]. Whether it is a minimally invasive surgery or development surgery, the recovery of low back muscle strength in patients with LDH after operation is very important. Early postoperative rehabilitation strengthens muscle strength and endurance, maximizes compensatory effects, and restores the spinal stabilisation system to reduce spinal instability caused by muscle atrophy [30, 31]. The incidence of complications can be reduced such as low back pain, dyskinesia, and muscle weakness. The timing of sports rehabilitation after open surgery is still clinically controversial. Therefore, clinical rehabilitation scholars began to study the effect and feasibility of rehabilitation exercise within 3 months after operation [32]. Postoperative patients with minimally invasive or no internal fixation can start rehabilitation training immediately after operation, and functional rehabilitation training as early as possible can more effectively reduce the occurrence of complications [33–35]. In patients with postoperative internal fixation, early rehabilitation may increase the risk of loosening of the implants. Because they are not fixed to the bone for a short period of time, the choice of exercise modality becomes particularly important. Different forms of exercise are subjected to different stress loads and early overloads or movements with a greater range of motion [36]. This would increase the risk of loosening of the internal fixation and breakage of the internal fixation due to excessive pressure. If this occurs, it will lead to surgical failure and significant cost to the patient. When choosing the exercise method, we should choose the exercise program with controllable strength and avoid a large range of motion in the spine as far as possible. According to the type, quantity, and segment of internal fixation, the risk coefficient of early postoperative rehabilitation is also very different. The more the number of internal fixation and the more complex the etiology before operation, the risk of fatigue fracture of internal fixation due to excessive stress in early postoperative rehabilitation training is also increased [37]. It was found that the load of 2 vertebral body fixation was higher than that of 3 vertebral body internal fixation under bending or axial load. The load of the two fixed segments is 49% of that of the three fixed segments in the tensile load test. In the end screw experiment, the results were the opposite with 2 internal fixation loads being smaller than 3 internal fixations in flexion and lateral bending [38]. There was no significant difference between compression test and tension test. The load of surgical implants varies with the change of human posture. According to the results of Rohlmann and other studies, it is concluded that when people lie on their backs or slopes, the pressure on the implants is the least compared to standing and exercise in the supine or oblique posture which can be considered to reduce the risk of loosening or breaking the implants. The load of internal fixation in sitting position is less than that in standing position. When the posture changes, the internal fixation load varies according to different posture. The internal fixation load such as simple sitting up and side bending is 1.11-1.20 times that of standing, and the upper body is increased when there is no weight in the standing position [39]. The results have suggested that the maximum load of internal fixation is 1.28 times that of walking and the minimum risk load to avoid fatigue fracture of pedicle screw is 1.1 times less than that of standing position. In the early stage, the functional exercise of patients should be guided step by step, starting from the axial turn of the lying position, gradually to sit up in the lateral position, sit up in the lateral position and stand with the aid of a walker, and then walk with the aid of a walker after standing for a certain period of time. When the patient can walk flexibly with the aid of the walker, he can walk independently without the aid of the walker. The early functional exercise of low back muscle adopts isometric contraction training to isotonic contraction training step by step, which can effectively reduce the risk of loosening or fracture of internal fixation after operation. Referring to the previous literature, it is found that it is safe and effective to start rehabilitation within 3 months after operation. This is mainly because the theory that prolonged bed rest leads to useless atrophy of the lumbar extensor muscles has been accepted by most scholars. Prolonged postoperative bed rest does not help the injured muscles to recover but rather causes the uninjured muscles to atrophy faster due to lack of active contraction and thus loss of innervation [40]. In addition, long-term immobilization aggravates the muscle contractile dysfunction, which is easy to cause local blood stasis in the venous system, increase capillary bed pressure, relatively reduce blood flow, and aggravate the accumulation of blood and lymph in the muscle, so that the muscle cannot get adequate blood supply and oxygen and muscle nutrition decline, resulting in more adverse effects on the stable system injured by surgery. The utilization of muscle glycogen will also decrease due to the decrease of muscle activity, resulting in the accumulation of lactic acid and muscle metabolites, accelerating fat infiltration instead of muscle, and further aggravating muscle atrophy. It is worth noting that lying in bed for a long time will accelerate the aging of the low back muscles; this atrophy may last for a long time and is not easy to recover [41].

At present, relying solely on the traditional health intervention model is not effective in improving patients' bad life behavior. Additionally, the intervention project is guided by health education, and health promotion theory has attracted more and more attention from all walks of life. Protective motivation intervention model is a new type of health intervention model formed under the guidance of the theory of protective motivation [42]. In recent years, this theoretical intervention model has been applied in preventing children from falling, reducing tobacco use among adolescents, and promoting nutrition improvement for the middle-aged and elderly and other fields and achieved good outcomes. Protective motivation theory is an extension and expansion of health theory, which focuses on the relationship between the environment and individual behavior and can effectively determine the level of health threat and susceptibility, reduce risk factors, and improve the quality of life of patients. In recent years, this theory has been applied in more and more fields. The theory of protective motivation is highly scientific and comprehensive, which can deeply analyze the internal mechanism of behavior change and promote the establishment of healthy behavior [43]. It can explain and predict the possibility of people accepting healthy behavior, improve the disease and surgical awareness of patients with lumbar disc herniation, mobilize patients' enthusiasm for treatment and improve doctor-patient relationship, and then improve the compliance behavior of patients in order to achieve the therapeutic effect. In addition, the theory of protective motivation combines the aspects of reaction cost, external reward, severity, response efficiency, susceptibility, self-efficacy, and internal return to deepen the concept of nursing and help patients build treatment confidence and alleviate their bad emotions. It can improve patients' treatment compliance and promote the recovery of patients' symptoms. There are some limitations in this study. First, the sample size of this study is not large, and it is a single-center study, so bias is inevitable. In future research, we will carry out multicenter, large-sample prospective studies, or more valuable conclusions can be drawn.

To sum up, the use of protective motivation intervention rehabilitation model can reduce the cognitive level of patients with lumbar disc herniation, reduce pain, improve their lumbar function, and then improve the quality of life of patients. This intervention program is worth popularizing.

## Figures and Tables

**Figure 1:** Comparison of JOA score between the two groups. Note: the JOA scores of the two groups at 1 month, 2 months, and 3 months after intervention were significantly lower than those before intervention (*P* < 0.05). After 1 month, 2 months, and 3 months after the intervention, the JOA scores of the research group were lower than those of the control group with the statistically significant difference (*P* < 0.05).

**Figure 2:** Comparison of RMDQ scores between the two groups. Note: the RMDQ scores of the two groups at 1 month, 2 months, and 3 months after intervention were significantly lower than those before intervention (*P* < 0.05). After 1 month, 2 months, and 3 months after the intervention, the RMDQ scores of the research group were lower than those of the control group, and the difference was statistically significant (*P* < 0.05).

**Table 1:** The scores of disease knowledge between the two groups ($\bar{x}\pm s$, points).

Group	*N*	Before intervention	One month after intervention	2 months after intervention	3 months after intervention
C group	70	13.53 ± 3.21	14.53 ± 4.53^a^	16.53 ± 4.66^ab^	18.53 ± 4.12^abc^
R group	70	13.24 ± 3.11	19.32 ± 3.41^a^	24.64 ± 3.64^ab^	27.54 ± 5.22^abc^
*t*		0.542	7.068	11.474	11.335
*P*		>0.05	<0.01	<0.01	<0.01

Note: ^a^compared with before intervention, *P* < 0.05; ^b^compared with 1 month after intervention, *P* < 0.05; ^c^compared with 2 months after intervention, *P* < 0.05.

**Table 2:** VAS scores between the two groups ($\bar{x}\pm s$, points).

Group	*N*	Before intervention	One month after intervention	2 months after intervention	3 months after intervention
C group	70	7.54 ± 2.53	4.64 ± 2.12^a^	2.16 ± 1.33^ab^	1.15 ± 0.56^abc^
R group	70	7.61 ± 2.56	6.21 ± 2.56^a^	5.35 ± 1.68^ab^	4.63 ± 1.57^abc^
*t*		0.162	3.951	12.455	17.467
*P*		>0.05	<0.01	<0.01	<0.01

Note: ^a^compared with before intervention, *P* < 0.05; ^b^compared with 1 month after intervention, *P* < 0.05; ^c^compared with 2 months after intervention, *P* < 0.05.

**Table 3:** PBPI scores between the two groups ($\bar{x}\pm s$, points).

Group	*N*	Before intervention	One month after intervention	2 months after intervention	3 months after intervention
C group	70	17.53 ± 2.31	15.24 ± 2.52^a^	13.83 ± 2.24^ab^	12.52 ± 2.15^abc^
R group	70	16.89 ± 2.33	10.42 ± 2.12^a^	6.53 ± 1.53^ab^	4.31 ± 1.03^abc^
*t*		1.632	12.245	22.515	28.812
*P*		>0.05	<0.01	<0.01	<0.01

Note: ^a^compared with before intervention, *P* < 0.05; ^b^compared with 1 month after intervention, *P* < 0.05; ^c^compared with 2 months after intervention, *P* < 0.05.

**Table 4:** SF-36 scores between the two groups ($\bar{x}\pm s$, points).

Group	*N*	Group		Psychological function		Social function		Mental health	
		Before intervention	After intervention	Before intervention	After intervention	Before intervention	After intervention	Before intervention	After intervention
C group	70	72.42 ± 5.53	83.63 ± 6.53^a^	77.52 ± 5.31	87.53 ± 6.35^a^	81.24 ± 6.42	90.12 ± 6.38^a^	80.31 ± 6.42	92.35 ± 7.14^a^
R group	70	73.04 ± 4.67	89.75 ± 6.14^a^	76.42 ± 5.24	94.51 ± 6.66^a^	80.21 ± 6.36	94.52 ± 6.74^a^	81.25 ± 6.26	96.41 ± 7.35^a^
*t*		0.716	5.712	1.233	6.346	0.953	3.966	0.866	3.314
*P*		>0.05	<0.01	>0.05	<0.01	>0.05	<0.01	>0.05	<0.01

Note: ^a^compared with before intervention, *P* < 0.05.

## Data Availability

No data were unavailable due to the privacy of patients.
